# Hypoxia-Activated PI3K/Akt Inhibits Oxidative Stress via the Regulation of Reactive Oxygen Species in Human Dental Pulp Cells

**DOI:** 10.1155/2019/6595189

**Published:** 2019-01-09

**Authors:** Fei Liu, Xin Huang, Zhenhua Luo, Jingjun He, Farhan Haider, Ci Song, Ling Peng, Ting Chen, Buling Wu

**Affiliations:** ^1^Department of Stomatology, Nanfang Hospital, Southern Medical University, Guangzhou 510515, China; ^2^College of Stomatology, Southern Medical University, Guangzhou 510515, China; ^3^International Medical Center, Guangdong Second Provincial General Hospital, Guangzhou 510317, China; ^4^Department of Stomatology, Guangzhou Women and Children's Medical Center, Guangzhou Medical University, Guangzhou 510623, China; ^5^Division of Gastroenterology, Hepatology and Nutrition, Cincinnati Children's Hospital Medical Center, Cincinnati, Ohio 45229, USA; ^6^Department of Biochemistry, Zhongshan School of Medicine, Sun Yat-sen University, Guangzhou 510080, China

## Abstract

In order to use stem cells as a resource for tissue regeneration, it is necessary to induce expansion *in vitro*. However, during culture, stem cells often lose functional properties and become senescent. Increasing evidence indicates that hypoxic preconditioning with physiological oxygen concentration can maintain the functional properties of stem cells *in vitro*. The purpose of the current study was to test the hypothesis that hypoxic preconditioning with physiological oxygen concentration can maintain the functional properties of stem cells in culture by reducing oxidative stress. *In vitro* studies were performed in primary human dental pulp cells (hDPCs). Reduced levels of oxidative stress and increased cellular “stemness” in response to physiological hypoxia were dependent upon the expression of reactive oxygen species (ROS). Subsequently, RNA-sequencing analysis revealed the increased expression of phosphoinositide 3-kinase (PI3K)/Akt signaling in culture, a pathway which regulates oxidative stress. Furthermore, we found evidence that PI3K/Akt signaling might affect intracellular ROS production by negatively regulating expression of the downstream protein Forkhead Box Protein O1 (FOXO1) and Caspase 3. Collectively, our data show that the PI3K/Akt pathway is activated in response to hypoxia and inhibits oxidative stress in a ROS-dependent manner. This study identified redox-mediated hypoxic preconditioning regulatory mechanisms that may be significant for tissue regeneration.

## 1. Introduction

Tissue regeneration requires the implantation of cellular adaptations to a wounded environment featuring a lesion. Because of their highly proliferative, multidifferentiation potential and low immunogenicity, hDPCs are considered to represent a promising source of stem cells for regenerative medicine and engineering tissue [1, 2]. However, stem cells become aged during *in vitro* expansion, and the transplantation environment can often be extremely harsh for such cells, thus representing a significant challenge for regenerative medicine. An increasing number of studies pertaining to pretreatment strategies have attempted to improve the *ex vivo* expanded microenvironment and thus facilitate implantation, homing, and survivability [3–6]. Hypoxic preconditioning (HP) is a direct and effective strategy in which to promote the *in vivo* survival and differentiation of transplanted stem cells; this is a vital factor for the success of stem cell-based tissue regeneration [7–9].

In recent years, hypoxia has also been found to play an important role in a number of physiological processes. Different levels of hypoxia are associated with various physiological behaviors and can regulate signal transduction in stem cell proliferation and differentiation during embryogenesis [10–12]. One of the advantages of living in a hypoxic niche is that stem cells can maintain a slowly circulating proliferation rate while avoiding tissue-related oxidative stress [13]. Essentially, all cells that undergo aerobic metabolism can produce ROS. This oxide can destroy DNA stability and induce oxidative stress in cells [13, 14]. The response of cells to ROS is highly dependent on other factors such as cell phenotype, cell differentiation status, or another stimulus state [15]. For example, hematopoietic stem cells (HSCs) have lower levels of ROS than differentiated hematopoietic cells [12]. There is a fine balance between ROS and hypoxia.

Physiological oxygen tension varies from 1% to 14% and is much lower when culturing *in vitro* [13]. Although there is no definitive experimental data for the measurement of physiological oxygen concentration in human dental pulp, a previous study using a rat animal model found that the oxygen concentration of incisor pulp tissue was approximately 3% [16]. The present literature relating to the effect of hypoxia on phenotypic changes in hDPCs shows that different oxygen-dependent concentrations are used for the treatment of hDPCs and that such changes are variable [17], especially in terms of cell differentiation and proliferation [18–20]. However, experiments have shown that the angiogenic ability of dental pulp cells after HP is significantly higher than that under normoxic conditions [21]. In addition, HP-treated cells exhibit increased levels of exosome secretion, which are effective in enhancing effector cell osteogenic and angiogenic capacity [22]. Contradictory reports of hypoxic preconditioning may be due to various conditions such as the degree of hypoxia, different cell lines, culture time, and donor's age.

To test the hypothesis that HP within the physiological range of oxygen concentration can maintain cell stemness by reducing oxidative stress in hDPCs, we investigated the effect of HP on the properties of oxidative stress and stemness. Our findings reveal that HP may effectively modulate oxidative stress in hDPCs via the PI3K/Akt pathway.

## 2. Material and Methods

### 2.1. Cell Identification and Culture

First, hDPCs were collected from the pulp tissues of extracted third molars (patient age: 15 to 25 years old). Cells from the first to the fifth passages were used in this study. All patients were informed, agreed to participate, and signed informed consent forms for scientific experiments involving tooth extraction. The study protocol was performed according to a standard protocol approved by the Ethics Committee of the Guangdong Provincial Second People's Hospital. Multidifferentiation of hDPCs was performed according to a procedure described previously [23]. Once cells had reached 80% confluency, hDPCs were allowed to differentiate in an osteogenic, chondrogenic, and adipogenic induction medium. The induction medium was changed after every 2 days until the differentiated cells were harvested.

### 2.2. Cell Preconditioning

Hypoxic preconditioning was established using the Hypoxia Chamber 27310 (Stemcell, Vancouver, CA). All hypoxia experiments were performed at 3% oxygen concentration. The preconditioning of reoxygenation was first carried out under hypoxia for 2 d and then returned to normoxia for the remaining experimental duration. hDPCs were cultured in different oxygen concentrations and treated with 0.5 mM/L N-acetyl-L-cysteine (NAC), 100 *μ*M/L hydrogen peroxide (H_2_O_2_), and 10 *μ*M/L LY294002. NAC and LY294002 were provided by Selleck, Houston, USA. H_2_O_2_ was provided by Nanjing Jiancheng, China.

### 2.3. Cell Counting Kit 8 Assay

The viability of hDPCs was assessed by the cell counting kit 8 (CCK8, Dojindo, Kyushu island). Cells were seeded at a concentration of 2000 cells per well, and the culture procedure was performed according to the manufacturer's instructions. Optical density was measured by absorbance at 450 nm using an ELx800 microplate reader (BioTek Instruments Inc., Vermont, USA).

### 2.4. Cell Cycle Analysis

After culturing in different oxygen atmospheric environments, cells were harvested and fixed with 70% alcohol at 4°C overnight. The supernatant was completely removed and cells incubated in propidium iodide for 30 minutes at room temperature, in the dark. Cells were then analyzed by flow cytometry using a flow cytometer (Becton Dickinson, San Diego, CA).

### 2.5. Analysis of Cell Surface Markers

After pretreatment for 2 d, cells were washed and resuspended in staining medium (PBS containing 1% fetal bovine serum), then labelled with monoclonal antihuman STRO-1-FITC, CD34-PE, DO105-PE, CD133-PE, and OCT4-PE (Chemicon, Temecula, CA) for 30 minutes on ice. Cells were then washed twice and resuspended in stain buffer for analysis by flow cytometry.

### 2.6. Colony-Forming Assay

Cells were digested to a single-cell suspension, and 1000 cells were plated in a 6-well plate. After pretreatment for 10 days, hDPCs were fixed with 4% paraformaldehyde for 30 min at room temperature and then stained by crystal violet for 15 min. Cells were then observed under an optical microscope, and the number of colonies with more than 50 cells was counted.

### 2.7. Measurement of ROS Level

Levels of intracellular ROS were measured with a ROS assay kit (Nanjing Jiancheng, China) after treatment with different culture conditions. Cells were then stained with dihydrodichlorofluorescein diacetate (DCFDA) at a concentration of 10 *μ*M for 45 min. Individual cells were measured by flow cytometry; 10,000 cells were analyzed for each sample.

### 2.8. Measurement of Apoptosis Ratio

An apoptosis assay was conducted using a KeyGEN apoptosis detection kit (KeyGEN Biotech Co., Nanjing, China) following the manufacturer's protocol. After pretreatment in each group, cells were collected and resuspended in a 10x binding buffer. Cells were then incubated with annexin V-FITC/propidium iodide (PI). Finally, samples were analyzed by flow cytometry; 10,000 cells were analyzed for each sample.

### 2.9. Measurement of Antioxidative Enzyme Activity

Cells were cultured in normoxic and hypoxic conditions. Levels of superoxide dismutase (SOD), catalase (CAT), and glutathione peroxidase (GSH-PX) were all determined by commercial assay kits (Nanjing Jiancheng, China).

### 2.10. Enzyme-Linked Immunosorbent Assay (ELISA)

Cells were cultured in normoxic and hypoxic conditions. Levels of IL-6 (interleukin-6) and IL-*β*1 (interleukin-*β*1) in culture supernatants were then assayed by enzyme-linked immunosorbent assay (ELISA; BioLegend) according to the manufacturer's instructions.

### 2.11. Western Blotting Assay

Cells were first collected using standard procedures. Total protein was then measured by the BCA Protein Assay Kit (Pierce Biotechnology, Rockford, IL), loaded for sodium dodecyl sulfate gel electrophoresis and transferred onto polyvinylidene fluoride membranes (Millipore, Billerica, MA). The membranes were then blocked with skimmed milk at room temperature for 1 hour and incubated at 4°C overnight with primary antibodies against HIF-1*α* (Santa Cruz, California, USA), PI3K (Abcam, Cambridge, UK), p-PI3K(Abcam, Cambridge, UK), Akt (Abcam, Cambridge, UK), p-Akt (Abcam, Cambridge, UK), Caspase 3 (Abcam, Cambridge, UK), and FOXO1 (Cell Signaling, Boston, USA). Total levels of GAPDH were used as a control. Densitometric analysis was performed using ImageJ Plus software (NIH, USA), and relative protein expression was calculated after normalization of the target total protein.

### 2.12. Bioinformatic Analysis

RNA-seq: hDPC gene expression profiling was performed using RNA deep sequencing by Annoroad Gene Technology Co. Ltd. (Beijing, China). Paired-end RNA-seq reads were mapped to the reference human genome (hg19) using HISAT2 (version 2.0.4). Read counts were calculated by HTSeq. Differential expression analysis was performed by DESeq2. For differential expression analysis, the fold-change cutoff was set at 2 or higher. Benjamini–Hochberg false discovery rate-adjusted *p* value less than 0.05 was considered statistically significant. Kyoto Encyclopedia of Genes and Genomes (KEGG) pathway analysis: 2-fold change, FDR-adjusted *p* value less than 0.05 genes was subjected to KEGG pathway analysis using ToppFun (https://toppgene.cchmc.org/enrichment.jsp) in the ToppGene toolbox (https://toppgene.cchmc.org/). Protein-protein interaction network analysis: protein-protein interactions among differentially expressed genes were retrieved from the STRING v10 database. The interaction network was generated by Cytoscape. Graph plotting: volcano plots and bar plots were generated by the ggrepel R package and GraphPad Prism 5, respectively. The heatmap was created by GENE-E software using expression profiles of 2-fold-changed genes in PI3K-Akt signaling pathways as input. The expression levels are displayed as *z*-score normalized counts per million (CPM) mapped fragment value. CPM values of each gene were *z*-score transformed normalized across all samples.

### 2.13. Statistical Analysis

All results are expressed as means ± standard deviation (SD). Statistical significance was determined using a *t* test or one-way analysis of variance (ANOVA). When *p* < 0.05, the difference was considered to be statistically significant.

## 3. Results

### 3.1. Derivation of hDPCs from Mesenchymal Tissue with Multipotential Differentiation Potential

To investigate the multidirectional differentiation potential of hDPCs, we first established hDPCs from pulp tissues of extracted third molars (patient age: 15 to 25 years). Cell surface marker identification experiments showed that hDPCs were derived from mesenchymal tissue and expressed mesenchymal specific surface markers (Figure 1(a)). Multidirectional differentiation experiments showed that hDPCs could differentiate into osteogenesis, cartilage, and adipocytes and express their corresponding specific markers (Figure 1(b)). Collectively, these data proved that hDPCs exhibit multidirectional differentiation potential.

### 3.2. HP Improves the Stemness of hDPCs

To investigate cellular responses to hypoxia in hDPCs, we investigated stemness and proliferation. The specific expression of hypoxia-inducible factor 1-alpha (Hif-1*α*) was enhanced when the hDPCs were under hypoxic conditions. The expression of HIF-1*α* reached maximal expression at 1 d, then slowly decreased (Figure 2(a)). The CCK-8 assay results revealed that HP treatment decreased cell viability for a certain period of time. Compared with the control group, the viability of the hypoxic group was slightly decreased. The late change of the reoxygenation group was similar to that of normoxia (Figure 2(b)). However, cell cycle experiments showed that HP can reduce the proportion of hDPCs in the G0/G1 phase and increase the proportion of cells in the S phase (Figure 2(c)) The ability for cell self-renewal was significantly improved after long-term hypoxia treatment (Figure 2(d)). Moreover, microscopical analysis showed that cells were smaller in size under hypoxic culture than under normoxia. The expression of the cell surface markers CD133 and CD34 was increased, while that of CD105 and OCT4 did not change significantly (Figure 2(e)). These results demonstrated that HP improves the stemness of hDPCs, especially during long-term processing.

### 3.3. HP Reduces Oxidative Stress in hDPCs

A ROS activity assay found that hypoxia reduced the release of ROS in hDPCs. Mean ROS activity in the reoxygenation group (hypoxia 2 d + normoxia 1 d) was higher than that in the hypoxic group but lower than that in the normoxia group (Figure 3(a)). After hypoxia treatment, expression of the inflammatory cytokine IL-6 and IL-1*β* was not statistically significant (Figure 3(b)). The proportion of apoptosis was lowest in the hypoxia group (Figure 3(c)). In the antioxidant enzyme experiment, HP-treated hDPCs showed an increased level of expression of the antioxidant enzyme GSH-PX, although there was no significant change in the levels of SOD and CAT (Figure 3(d)). These results indicated that HP slightly reduced oxidative stress in hDPCs.

### 3.4. Bioinformatic Analysis Revealed Activation of the PI3K/Akt Pathway under Hypoxic Conditions

To better understand the molecular mechanisms underlying hypoxia-induced changes, we performed whole transcriptome RNA-seq analysis in hDPCs. Differential expression analysis identified 1271 upregulated genes and 559 downregulated genes after hypoxia for 48 hours compared to normoxia. Importantly, we observed numerous protein-protein interactions among proteins encoded by differentially expressed genes (Supplementary Figure 1). These proteins formed a condensed interaction network with multiple hypoxia-induced proteins, such as ENO2, as hubs. To explore cellular signaling further, we conducted Kyoto Encyclopedia of Genes and Genomes (KEGG) pathway analysis with the ToppGene tool. Downregulated genes in hypoxia showed enrichment of protein synthesis and metabolic pathways while glycolysis and cell cycle-related pathways were enriched in upregulated genes (Figures 4(a) and 4(b)). As expected, the HIF-1 signaling pathway was one of the top 10 enriched pathways in hypoxia (Figure 4(b)). We observed that the PI3K/Akt signaling pathway was also activated in hypoxia (Figure 4(b)). Notably, a substantial number of genes (32 genes) in the PI3K/Akt signaling pathway, including the cell cycle regulator, CDK2, are increased in hypoxia. Interestingly, we also found that 12 genes in this pathway are downregulated in hypoxia. This data seems to be paradoxical as we observed two sets of genes with opposite expression profiles in the same pathway, which also prompted us to experimentally investigate function of the PI3K/Akt pathway in hypoxia. Additionally, these data suggest that hDPCs may enhance cell proliferation and antioxidative stress in response to hypoxia stress.

### 3.5. PI3K/Akt Signaling Is Involved in the Regulation of Cellular Redox Status under Hypoxic Conditions

Given the essential roles of PI3K/Akt signaling in the response to hypoxia, we next examined whether inhibition of this pathway could change cellular phenotypes. LY294002, an inhibitor of the PI3K/Akt pathway, could enhance the expression of ROS and the apoptosis ratio in hDPCs (Figures 5(a) and 5(b)), although LY294002 has the same effect on ROS and apoptosis under normoxia or hypoxia. However, under hypoxia condition, the differences within the group are more obvious. These results indicate that HP can effectively regulate the production of ROS in hDPCs through the PI3K/Akt pathway. Inhibitor-treated cells showed reduced expression of the inflammatory cytokine IL-6 and increased levels of IL-1*β*; however, there was no significant difference between hypoxia and normoxia (Figure 5(c)). It is suggested that the PI3K/Akt pathway may not be involved in the release of these two inflammatory factors pass by changed oxygen concentration. The expression of the antioxidant enzymes SOD and CAT did not change significantly, while the expression of GSH-PX decreased, indicating that the PI3K/Akt pathway is partially involved in the regulation of antioxidant enzyme expression levels (Figure 5(d)). Expression of phosphorylated PI3K and Akt was higher in the hypoxia group. The expression of phosphorylated PI3K and Akt in the NAC group was higher than that in the H_2_O_2_ and LY294002 group. The expression of Caspase 3 was similar to that of FOXO1 but in stark contrast to the expression of p-PI3K and p-Akt (Figure 5(e)). These findings are consistent with results arising from the bioinfomatic analysis in that the treatment of hDPCs with HP activates phosphorylation of the PI3K/Akt pathway. The degree of phosphorylation in the PI3K/Akt pathway was decreased in cells under oxidative stress, and the effect of the inhibitor LY29004 was similar to H_2_O_2_. Moreover, Caspase 3 and FOXO1 may act downstream of the PI3K/Akt pathway, regulating the stress state of cells. PI3K/Akt signaling may affect intracellular ROS production by reverse regulating expression of the downstream protein FOXO1 and Caspase 3.

## 4. Discussion

Human dental pulp cells, as an adult stem cell, have not yet achieved widespread clinical applications, mainly because their source is limited, and because there have been issues with expansion and senescence during *in vitro* culture. Physiological hypoxia stimulates cells to adapt and increase their levels of glycolytic metabolism, thus reducing activity of the tricarboxylic acid (TCA) cycle and oxidative phosphorylation, which helps to reduce mitochondrial ROS production [10, 24]. ROS acts as a signaling molecule with low levels of homeostatic function or as a deleterious factor associated with high levels of tissue damage [10].

In the present study, we demonstrated that the HP treatment of hDPCs have a significant impact on cell self-renewal by reducing cell apoptosis ratio and ROS expression, while increasing colonial formation ability and the expression of the antioxidant enzyme GSH-PX. CD133, CD105, and OCT4 are considered to represent positive markers for mesenchymal stem cells. Evidence suggests that hypoxic preconditioning enhances the expression of these markers. In our experiment, the expression of CD133 was increased slightly after 2 days of hypoxic preconditioning. At the same time, the expression of CD34, a marker associated with hematopoietic function, was not statistically different and did not affect the qualitative properties of the hDPCs. The slight increase in expression may be related to a hypoxic function that promotes angiogenesis. In general, short-term hypoxic pretreatment (2 d) compared with long-term pretreatment (10 d) did not achieve a significant impact on cell phenotype.

In this study, oxygen-sensitive transcriptional programs in hDPCs were analyzed by bioinformatics tools, and their gene expression profiles were determined. Results showed that a variety of HIF-controlled genes, and genes encoding glycolytic enzymes and pentose phosphatase, were upregulated under two different low oxygen tension culture conditions. These experiments demonstrate the importance of using physiological hypoxic conditions, which mimic the anile environment of hDPCs to maintain pluripotency. Our data showed that the expression of PI3K/Akt was enhanced under hypoxic conditions. Many studies have reported that PI3K/Akt signaling can regulate the ROS expression, as well as the pathways involved in cellular oxidative stress [15, 25].

Further experimental results showed that the ratio of apoptotic cells and expression level of ROS increased after addition of the inhibitor LY294002. There was no significant change in the expression of the antioxidant enzymes and inflammatory cytokines, indicating that PI3K/Akt is not involved in the regulation of expression. Modulation of the expression of antioxidant enzymes and inflammatory cytokines may involve another molecular pathway simultaneously, such as APE-1/Ref-1 [26, 27] and Nrf2 signaling [28, 29]. However, there was significant change in GSH-PX levels, indicating that PI3K/Akt is involved in the upregulation of expression. Phosphorylated PI3K (p-PI3K) and Akt (p-Akt) expression increased and decreased after adding NAC and H_2_O_2_, respectively. It is suggested that PI3K/Akt signaling is involved in the expression of ROS under hypoxia. It has been reported that HIF-1*α* cannot translocate to the nucleus when Akt is inhibited, demonstrating that this may play an important role in the upstream regulation of HIF-1*α* [30]. Our study emphasizes that there might be a necessary connection between the two signaling pathways. The FOXO subfamily of Forkhead transcription factors are important regulators of cell survival in response to a variety of stress-related stimuli, such as hypoxia, DNA damage, and nutrient-poor conditions. The results of western blotting confirmed that PI3K/Akt negatively regulates the expression of FOXO1, a downstream regulatory target of the PI3K/Akt pathway [31–33]. We speculate that FOXO1 may be involved in hypoxia. However, further in-depth studies are now needed to verify the relationship between FOXO1 and hDPCs under hypoxia.

In summary, we have discovered a novel redox-mediated molecular mechanism for regulating the self-renewal and differentiation potential of hDPCs. The PI3K/Akt pathway was activated in response to hypoxia and inhibited oxidative stress in a ROS-dependent manner.

## Figures and Tables

**Figure 1:** hDPC culture and identification of multidifferentiation ability: (a) identification of the mesenchymal stem cell surface markers CD105, CD133, and STRO1; (b) induced osteogenic, chondrogenic, adipogenic differentiation, and immunofluorescence staining of alkaline phosphatase (ALP), collagen type III (Col III), and lipoprotein lipase (LPL), respectively; nuclei were counterstained with 4′,6-diamidino-2-phenylindole (DAPI) (magnification 10 × 10).

**Figure 2:** HP changed the cell phenotypes of hDPCs after culture under normoxia, hypoxia, and reoxygenation: (a) western blot assay and quantitative analysis of the expression of HIF-1*α* under normoxia and hypoxia at 0 h, 4 h, 8 h, 12 h, 24 h, and 48 h of culture; (b) proliferation ability of hDPCs in each group; (c) flow cytometry and quantitative analysis of cell cycle distribution in hDPCs after 3 d of culture under different oxygen concentrations; (d) colony-forming units and quantitative analysis in hDPCs after 10 d of culture; (e) expression of the mesenchymal stem cell surface markers CD133, CD34, CD105, and OCT4 in each group. Statistical significance is shown as ^∗^ *p* < 0.05.

**Figure 3:** Effect of HP on oxidative stress in hDPCs after 3 d culture under normoxia, hypoxia, and reoxygenation: (a) HP-treated hDPCs were stained with 10 *μ*M DCFDA and analyzed by flow cytometry; (b) the expression of inflammatory cytokines in each group, as analyzed by ELISA; (c) flow cytometry and quantitative analysis of cell apoptosis ratio in each group; (d) activity of the antioxidant enzymes SOD, CAT, and GSH-PX in hDPCs during culture at different oxygen concentrations. Statistical significance is expressed as ^∗^ *p* < 0.05.

**Figure 4:** Differential expression analysis of hDPCs cultured between hypoxia and normoxia conditions: (a) top enriched pathways in downregulated genes of hypoxia condition; (b) top enriched KEGG pathways in upregulated genes of hypoxia condition; (c) heatmap shows expression of differentially expressed genes in the PI3K-Akt signaling pathway between hypoxia and normoxia conditions. Red indicates high expression, while blue indicates low expression.

**Figure 5:** Inhibiting the PI3K/Akt pathway changed the redox status of hDPCs after 2 d of culture under normoxia and hypoxia: (a) hDPCs were stained with 10 *μ*M of DCFDA and analyzed by flow cytometry; (b) flow cytometry and quantitative analysis of cell apoptosis ratio in different treatment groups; (c) levels of inflammatory cytokines secreted by each group, as determined by ELISA; (d) activity of the antioxidant enzymes SOD, CAT, and GSH-PX in hDPCs from each group; (e) western blot assay and quantitative expression of PI3K, p-PI3K, Akt, p-Akt, Caspase 3, and FOXO1 in different groups. Statistical significance is expressed as ^∗^ *p* < 0.05 versus *normoxia*; ^#^ *p* < 0.05 versus *control*.

## Data Availability

The RNA-seq data used to support the findings of this study are available from the corresponding author upon request.

## Supplementary Materials

Supplementary 1 Date 1: the fold changes of the ROS ratio and the detailed values of the statistical analysis, for both between-group and within-group comparisons.

Supplementary 2 Date 2: the fold changes of the apoptosis ratio and the detailed values of the statistical analysis, for both between-group and within-group comparisons.

Supplementary 3 Date 3: the fold changes and detailed values for the p-PI3K, p-Akt, Caspase 3, and FOXO1, for both between-group and within-group comparisons.

Supplementary 4 Figure 1: protein-protein interaction network analysis: protein-protein interactions among differentially expressed genes were retrieved from the STRING v10 database. Interaction network was generated by Cytoscape. We observed numerous protein-protein interactions among proteins encoded by differentially expressed genes. These proteins form a condensed interaction network with multiple hypoxia-induced proteins, such as ENO2, as hubs.
